RETRACTED

# Abnormal COX2 Protein Expression May Be Correlated with Poor Prognosis in Oral Cancer: A Meta-Analysis

**DOI:** 10.1155/2014/364207

**Published:** 2014-06-16

**Authors:** Zhi-Ming Wang, Jie Liu, Hong-Bo Liu, Ming Ye, Yu-Fei Zhang, Dong-Sheng Yang

**Affiliations:** ^1^Department of Stomatology, Shengjing Hospital of China Medical University, No. 36 Sanhao Street, Heping District, Shenyang 110000, China; ^2^Experimental Technology Center of China Medical University, No. 92 Beier Street, Heping District, Shenyang 110000, China; ^3^Department of Statistics, School of Public Health, China Medical University, Shenyang 110000, China

## Abstract

*Background.* The prognostic significance of COX2 for survival of patients with oral cancer remains controversial. Thus, the meta-analysis was performed in order to identify COX2 expression impact on prognosis of oral cancer. *Method.* Relevant literatures were searched using the following electronic databases without any language restrictions: Web of Science, the Cochrane Library Database, PubMed, EMBASE, CINAHL, and CBM. Version 12.0 STATA software (Stata Corporation, College Station, Texas, USA) was used for the current meta-analysis. Odds ratios (ORs) and hazard ratios (HRs) with their corresponding 95% confidence interval (95% CI) were also calculated to clarify the correlation between COX2 expression and prognosis of oral cancer. *Results.* Final analysis of 979 oral cancer patients from 12 clinical cohort studies was performed. The meta-analysis results show that COX2 expression in cancer tissues was significantly higher than those in normal and benign tissues (all *P* < 0.05). Combined HR of COX2 suggests that positive COX2 expression has a shorter overall survival (OS) than those of negative COX2 expression (*P* < 0.05). *Conclusion.* The meta-analysis study shows that elevated COX2 expression may be associated with the pathogenesis of oral cancer and with a worse prognosis in oral cancer patients.

## 1. Introduction

Oral cancer or mouth cancer is any cancerous tissue growth located in the oral cavity, which was regarded as the sixth most common diagnosed malignancy of all cancers worldwide [1]. Generally, over 90% of oral malignancies in the upper aerodigestive tract are squamous cell carcinomas, with the signs and symptoms of skin lesion, lump, ulcer, swallowing difficulty, and mouth sores [2]. As an important ongoing public health problem, the prevalence and morbidity of oral cancer were increased, with the number of an estimated 263,900 new invasive cases and 128,000 deaths in 2008 all over the world [3]. Furthermore, the majority of oral cancer patients had a significantly poor prognosis and the overall 5-year survival rate of oral cancer patients is less than 50% [3]. Indeed, oral cancer is known to be a complex and multifactorial disease which may be induced by the interaction of genetic and environmental factors [4, 5]. In the past few decades, tobacco use (both smoking and chewing) and alcohol consumption were considered to be the main risk factors for oral cancer, while age, gender, HPV infections, betel quid chewing, and other unhealthy lifestyles may also contribute to the pathogenesis and development of oral cancer [6, 7]. Recently, epidemiological study has revealed that cyclooxygenase-2 (COX-2) protein expression may be a biomarker for predicting the prognosis of oral cancer [8].

RETRACTED

The cyclooxygenase 2 (COX2), also known as prostaglandin-endoperoxide synthase 2 (PTGS2) in humans, is one of the two isoforms of COX that is the rate-limiting enzyme in the metabolic conversion of arachidonic acid to prostaglandins, including prostaglandin E2, a major mediator of inflammation and angiogenesis [9, 10]. Although its physiological role is not fully known, COX2 may function significantly in the inhibition of apoptosis and immune surveillance, the promotion of angiogenesis, the elevation of cancer invasiveness and metastasis, and the modulation of cell differentiation [11]. More importantly, COX2 is usually unexpressed under the normal circumstance in most cells, whereas increased levels are always found in response to inflammation reactions, growth factors, and tumor promoters [12]. In recent decades, overexpression of COX2 has been reported in various cancer types, such as those arising in the esophageal, breast, lung, colon, stomach, prostate, and urinary bladder [13–16]. On the contrary, selective COX2 inhibitors suppress growth of cells by inducing G0/G1, cell-cycle arrest, and cellular proliferation; thus apoptosis could have a reversed effect on the development and progression of cancers [17]. Similar to the results of the present study on the expression of COX2 and the pathogenesis of human tumors, previous reports have suggested a correlation between the expression of COX2 and the occurrence of oral cancer [18, 19]. In general, COX2 may initially stimulate angiogenesis and vascular endothelial cell growth that are essential in tumor growth and spread, promoting the production of prostaglandin E2 and cyclin-dependent kinase inhibitor P21 expression [20]. Due to its previous multiple functions, COX2 may participate in initiation, progression, invasion, and metastasis of cancer cells which are potential with clear prognostic implications and consequently contribute to the deterioration of human cancers [9]. In view of these above reasons, it was plausible to speculate that manipulation of serum levels of COX2 may be useful in the prediction of prognosis of oral cancer. In this regard, it may also be useful for the adoption of selective COX2 receptor-blocking agents in prevention of oral cancer by blocking initiation, progression, or metastasis of tumors [20]. In recent decades, several previous studies have confirmed that the elevated COX2 levels may be an indicator of biologically aggressive tumor prognosis based on its important role on tumor cells growth and metastasis [21, 22]; meanwhile other studies have also illustrated inconsistent results [8, 23]. Given the conflicting evidence on this issue, we conducted a meta-analysis of all available cohort studies to explore the associations between the serum level of COX2 and the prognosis in oral cancer patients.

RETRACTED

## 2. Materials and Methods

### 2.1. Literature Search

Web of Science (1945~2013), the Cochrane Library Database (Issue 12, 2013), PubMed (1966~2013), EMBASE (1980~2013), CINAHL (1982~2013), and the Chinese Biomedical Database (CBM) (1982~2013) were searched for relevant articles without any language restrictions. The keywords and MeSH terms we used in conjunction with a highly sensitive search strategy were as follows: [“Cyclooxygenase 2” or “Cyclooxygenase 2 Inhibitors” or “cyclooxygenase 2” or “cyclooxygenase 2 inhibitors” or “Cyclo-Oxygenase II” or “PTGS2” or “PTGS-2” or “Prostaglandin H Synthase-2” or “Cyclooxygenase-2” or “prostaglandin synthase 2” or “COX2 Inhibitors” or “cyclooxygenase-2 Inhibitors”] and [“Mouth Neoplasms” or “mouth neoplasms” or “oral neoplasm” or “oral cancer” or “mouth cancer” or “cancer of the mouth” or “oral carcinoma” or “mouth carcinoma” or “oral squamous cell carcinoma” or “OSCC”]. The above references of articles and reviews identified in the included articles were also performed to search for additional studies.

### 2.2. Inclusion and Exclusion Criteria

We collected all eligible articles about the relationship between COX2 and oral cancer in this meta-analysis. The study included in our meta-analysis should meet the following inclusion criteria: (1) COX2 expression is evaluated in the oral cancer tissues; (2) relationship is demonstrated between COX2 expression and oral cancer prognosis; (3) all COX2 expressions are examined by immunohistochemistry, and sufficient information about COX2 expression levels should be provided in the paper; (4) only the most complete single study was selected, if multiple studies investigated the same patients or potential overlapping patients. The exclusion criteria were also as follows: (1) letters, case reports, reviews, editorials, conference abstracts, and some non-English language articles; (2) papers that had no information of overall survival (OS) or that could not calculate the hazard ratios (HRs) about OS from the given information which were excluded.

RETRACTED

### 2.3. Data Extraction and Methodological Assessment

Using a standardized form, data extraction was performed independently by two authors from each included study. Two investigators reviewed all of researches that met the previous inclusion and exclusion criteria. Language of publication, publication year of article, the first author's surname, geographical location, design of study, total number of cases, sample size, the source of the subjects, detection method of protein expression, expression levels, TNM stage, clinicopathological parameters, immunohistochemical technique, COX2 expression, and patient survival results from each study were all documented. Study quality was assessed independently by two investigators, by means of reading and evaluating according to the Newcastle-Ottawa Scale (NOS) quality assessment scale [24]. Briefly, the overall star assessed three main categories in the following: (1) subject selection: 0~4; (2) comparability of subject: 0~2; (3) clinical outcome: 0~3. NOS scores ranged from 0 to 9; and a score ≥ 7 indicates a good quality. The total number of grades was accumulated at last, with more sensitivity reflecting a better methodological quality.

### 2.4. Statistical Analysis

We extracted and combined the data of COX2 expression and prognostic parameters associated with oral cancer from studies and made a meta-analysis. The Version 12.0 STATA statistical software (Stata Corporation, College Station, TX, USA) was employed in this study to achieve statistical analysis. For quantitative evaluation of OS results, OR and its corresponding 95% confidence interval (95% CI) were used to estimate the influence of COX2 expression on OS of oral cancer patients. The *Z* test was adopted to calculate the statistical significance of pooled HR and ORs. Heterogeneity among studies was estimated by Cochran's *Q*-statistic and *I* ^2^ tests [25]. A random-effect model was used when *Q*-test exhibits a *P* < 0.05 or *I* ^2^ test shows > 50%; otherwise, the fixed-effect model was used. We also make use of subgroup analyses to explore sources of heterogeneity. For the purpose of evaluating the influence of single studies on the overall estimate, a sensitivity analysis was performed. Funnel plots and Egger's linear regression test were applied to explore the potential publication bias [26].

## 3. Result

### 3.1. Characteristics of Included Studies

Initially, the highly sensitive search strategy identified 264 articles. After a rough review of the titles and abstracts of all the articles, we further excluded 136 articles; The original search yielded a total of 264 papers related to the searched keywords. Through the step of screening the title and key words, 139 of these articles were excluded. Full-text from 125 articles was reviewed and an additional 111 trials were excluded, leaving 14 studies for further review. Of these, 2 were abandoned because of not supplying enough information (Figure 1). Another 2 studies were also excluded due to lack of data integrity (Figure 1). Eventually, 12 clinical cohort studies with a total of 979 oral cancer patients met our inclusion criteria for quantitative data analysis [8, 11, 18, 19, 21–23, 27–31]. There were 5 independent analyses focused on the prognosis of oral cancer, some of which were divided into two groups, including COX2-positive group (*n* = 157) and COX2-negative group (*n* = 254). Additionally, there existed 7 articles focused on protein expression of COX2, with a total of 419 oral cancer patients. As shown in Figure 2, the publication years of the eligible studies ranged from 2001 to 2013. Overall, 9 studies were conducted among Asians and the other 3 among Caucasians. Meanwhile, Envision, streptavidin-biotin-peroxidase complex (SABC), activity-based costing (ABC), streptavidin-peroxidase (SP), and Power Vision~(TM)-9000 (PV-9000) methods were utilized in the current meta-analysis. NOS scores of all included studies were ≥ 6. We summarized the baseline characteristics and methodological quality in Tables 1 and 2.

RETRACTED

### 3.2. Quantitative Data Synthesis

There were altogether 12 studies included focusing on the relationship between the expression of COX2 and the prognosis of oral cancer. The present meta-analysis indicated that the expression of COX2 protein in cancer tissues was significantly higher than those in normal and benign tissues (cancer tissues versus normal tissues: OR = 92.86, 95% CI = 53.61~160.84, *P* < 0.001; cancer tissues versus benign tissues: OR = 11.58, 95% CI = 6.68~20.08, *P* < 0.001, resp.). Considering the OS rate, our findings showed that COX2-positive group had a poor OS rate of oral cancer patients as compared to the COX2-negative group (HR = 2.23, 95% CI = 1.42~3.05, *P* < 0.001) (Figure 3).

Subgroup analysis based on sample size and detection method revealed that the expression of COX2 in the cancer tissues was correlated with the prognosis of oral cancer patients compared to those in the normal tissues and benign tissues in all these subgroups (all *P* < 0.05) (Figure 4). Furthermore, subgroup analyses by sample size and detection method also indicated that elevated expression COX2 protein was strongly linked to shorter OS of oral cancer patients in all these subgroups (all *P* < 0.05).

RETRACTED

A sensitivity analysis indicated that the overall pooled ORs and HRs could not be affected by single study (Figure 5). There was evidence for asymmetry in the funnel plots in the comparison of cancer tissues with normal and benign tissues; Egger's test showed a remarkable evidence of publication bias (all *P* < 0.05). However, with respect to the OS of oral cancer patients, there was no strong evidence in the funnel plots, and Egger's test also failed to present any evidence of publication bias (*t* = 0.78, *P* = 0.490) (Figure 6).

## 4. Discussion

The purpose of this meta-analysis was to investigate the association between the expression of COX2 protein and the clinical outcome in patients with oral cancer. Our results showed that there were significant correlations between COX2 protein expression and the recurrence-free or OS rate of oral cancer, suggesting that COX2 protein expression may have a prognostic significance in oral cancer. It is widely recognized that the use of nonsteroid anti-inflammatory drugs (NSAIDs) is closely correlated with a reduced risk of cancer [32]. Exactly, COX2 is the best known target of NSAIDs, which is considered as a critical rate-limiting enzyme in the arachidonic acid metabolism that is implicated in the biosynthesis of prostaglandins [33]. Moreover, prostaglandins have been documented to have a key role in creating a proangiogenic microenvironment in human tumors [34]. In addition, COX2 has been widely known as one of the crucial prognostic factors in carcinomas of the various organs [35, 36]. However, the importance of COX2 overexpression in oral cancer has not been fully described yet. As a matter of fact, the expression of COX2 protein was supported to be low or nondetectable in most human healthy tissues, whereas it can be highly stimulated in response to cell activation by proinflammatory cytokines, growth factors, hormones, or tumor promoters [18]. Most importantly, through different mediators, the alteration in COX2 expression may promote angiogenesis, increase cancer invasiveness and metastasis, regulate cell proliferation, and inhibit apoptosis and immune surveillance [37]. To be specific, the upregulation of COX2, at both mRNA and protein levels, may result in the enhanced synthesis of prostaglandins, increasing proliferative activity of neoplastic cells, and further accelerating angiogenesis and inhibiting immune surveillance; additionally, immunohistochemical overexpression of COX2 may thereby inhibit apoptosis and strength invasiveness [27]. In this regard, high expression levels of COX2-derived prostaglandin can be identified to be active in highly vascularized tumors, and in turn selective suppression of COX2 could lead to a decreased tumor growth because of the transformation in the neovasculature [23]. Therefore, we can postulate that the elevated expression of COX2 may have an important role in predicting the clinical outcome in oral cancer, and these many essential processes in carcinogenesis make COX2 an attractive therapeutic target. In consistence with our results, Cha et al. detected the expression of COX2 via immunohistochemistry analyses of 103 OSCC samples indicating that the upregulated COX2 expression in oral cell lines may be a possible prognostic parameter for reduced overall survival [19]. Similarly, Sakurai et al. also found that the expression of COX2 was related to lymph node metastasis and cell proliferative activity, as well as overall 5-year survival rate in oral carcinoma, and thereby this enzyme may be valuable in diagnostic and prognostic indices in oral carcinoma [11].

RETRACTED

Meanwhile, there did exist some limitations in the current meta-analysis. Firstly, due to a myriad of necessary information which cannot be successfully obtained, we did not take into account unpublished articles and abstract entirely. In this regard, our results did not implicate all the data from all trials to evaluate the impact of COX2 expression on the prognostic influence of oral cancer patients. Nevertheless, our meta-analysis managed to overcome limits of size or scope in individual studies to acquire more reliable and general information from each study. Secondly, the results of meta-analysis might slightly lack reliability to some extent since it is a retrospective study, which may induce potential publication bias. Particularly we picked up those eligible English studies only because of excluding parts of qualified studies based on language criteria. A third potential limitation is that our meta-analysis may still be underpowered to acquire original data from the included studies. Despite the above limitations, this is the first example of meta-analysis on the association of COX2 expression with the development of oral cancer. With the application of a statistical approach to combine the results from multiple studies in our meta-analysis and to achieve strong objectivity, all the research methods were carried out on strict inclusion and exclusion criteria. In addition, inconsistency of results was rigorously quantified and analyzed in our meta-analysis, which will finally contribute to a more reliable conclusion.

In conclusion, our results provide empirical evidence that COX2 protein expression may be negatively correlated with a worse prognosis in patients with oral cancer. Thus, expression of COX2 protein may be regarded as a prognostic factor for oral cancer patients relying on the present obtained data. However, larger clinical studies should be performed to explore the precise prognostic significance of COX2, and the determination of its nuclear and subcellular location should also be seriously considered in particular.

RETRACTED

## Figures and Tables

**Figure 1:** Flow chart shows study selection procedure. Twelve cohort studies were included in this meta-analysis.

**Figure 2:** The distribution of the number of topic-related literatures in electronic database over the last decade.

**Figure 3:** Forest plots for the relationships of abnormal COX2 protein expression with clinicopathological characteristics and prognosis of patients with oral cancer.

**Figure 4:** Subgroup analyses by sample size and detecting method of the relationships of abnormal COX2 protein expression with clinicopathological characteristics and prognosis of patients with oral cancer.

**Figure 5:** Sensitivity analysis of the summary odds ratio coefficients on the relationships of abnormal COX2 protein expression with clinicopathological characteristics and prognosis of patients with oral cancer.

**Figure 6:** Funnel plot of publication biases on the relationships of abnormal COX2 protein expression with clinicopathological characteristics and prognosis of patients with oral cancer.

**Table 1:** Main characteristics and methodological quality of all eligible studies on oral cancer prognosis.

First author	Year	Ethnicity	Number		Gender (M/F)	Age (years)	Method	Protein	NOS score
			Positive	Negative					
Haffner [23]	2012	Caucasians	27	64	74/22	64 (26~85)	Envision	COX2	8
Cha [19]	2011	Asians	39	64	77/26	—	Envision	COX2	6
Sakurai [11]	2007	Asians	61	19	—	—	SABC	COX2	6
Atula [18]	2006	Caucasians	20	45	44/21	58 (31~80)	ABC	COX2	7
Itoh [27]	2003	Asians	10	62	—	62.9 ± 13.0	Envision	COX2	6

M: male; F: female; NOS: Newcastle-Ottawa Scale; SABC: streptavidin-biotin-peroxidase complex; ABC: activity-based costing.

**Table 2:** Main characteristics and methodological quality of all eligible studies on oral cancer clinicopathological characteristics.

First author	Year	Ethnicity	Number			Gender (M/F)	Age (years)	Sample	Method	NOS score
			Tumor	Benign	Normal					
Li [8]	2013	Asian	38	33	10	21/17	25~72	Tissue	SP	8
Segawa [28]	2008	Asian	72	0	15	—	—	Tissue	SABC	6
Sawhney [29]	2007	Asian	107	0	15	85/22	—	Tissue	SABC	7
Cao [21]	2005	Asian	76	0	12	43/33	58 (36~83)	Tissue	PV-9000	8
Tang [30]	2003	Asian	27	0	4	—	—	Tissue	ABC	6
Sudbø [22]	2003	Caucasians	29	0	30	—	—	Tissue	ABC	6
Sakurai [31]	2001	Asian	30	0	15	—	—	Tissue	SABC	6
Sakurai [31]	2001	Asian	40	0	15	—	—	Tissue	SABC	6

M: male; F: female; NOS: Newcastle-Ottawa Scale; SABC: streptavidin-biotin-peroxidase complex; ABC: activity-based costing; SP: streptavidin-peroxidase; PV-9000: Power Vision-9000.
